The article "Identification of Cancer-Specific Methylation of Gene Combination for the Diagnosis of Bladder Cancer" was published in 2019. Journal: J Cancer.

# Identification of Cancer-Specific Methylation of Gene Combination for the Diagnosis of Bladder Cancer

**DOI:** 10.7150/jca.28192

**Published:** 2019-10-22

**Authors:** Ning Zhang, Siteng Chen, Lingfeng Wu, Yishuo Wu, Guangliang Jiang, Jialiang Shao, Lixin Chen, Jishan Sun, Rong Na, Xiang Wang, Jianfeng Xu

**Affiliations:** 1 Department of Urology, Ruijin Hospital, Shanghai Jiao Tong University School of Medicine, Shanghai, China;; 2 Department of Urology, Shanghai General Hospital, Shanghai Jiao Tong University School of Medicine, Shanghai, China;; 3 Department of Urology, Songjiang District Central Hospital, Shanghai, China;; 4 Department of Urology, Huashan Hospital, Fudan University, Shanghai, China;; 5 Department of Urology, Shengzhen Second People's Hospital, Guangdong, China.; 6 Program for Personalized Cancer Care, Northshore University HealthSystem, Chicago, IL 60201.

**Keywords:** bladder cancer, urine, DNA methylation, biomarker

## Abstract

Here we conducted an evidence-based study in developing and validating a urinary biomarker combination of gene methylation assays in patients with hematuria. A number of 99 urine samples were obtained and detected from Chinese patients with hematuria. The Cancer Genome Atlas cohort with methylation (HM450) beta-values and clinical data of 412 bladder cancer and 21 matching normal tissue was included as a validation series. A risk score formula was then developed and calculated by the targeted genes, weighted by their estimated regression coefficients from the multivariable binary logistic regression analyses, and evaluated by receiver operating characteristic (ROC) curves analysis. The combination assay of *HOXA9*, *ONECUT2*, *PCDH17*, *PENK*,* TWIST1*,* VIM* and *ZNF154* was singled out according to the results of multivariate logistic regression analysis. The higher probability of DNA methylation of all the selected 7 genes was found in bladder cancer group than the control group. Remarkable higher DNA methylation beta-values of all the selected 7 genes were also displayed in bladder cancer tissues compared with their matching normal bladder tissues. And the AUC value of our risk score model were 0.894 and 0.851 in respective cohort, revealing highlighted predictive value of our risk score model on bladder cancer diagnosis. In conclusions, a urinary combined methylation assay of *HOXA9*, *ONECUT2*, *PCDH17*, *PENK*,* TWIST1*,* VIM* and *ZNF154* displayed accurate prediction of bladder cancer in hematuria patients, which provided the guidance for the patients at early stage tumor and during the follow-up after operation. Of course, prospective study based on a hematuria cohort with a large sample size should be conducted to validate these findings in the future.

## Introduction

As a highly aggressive carcinoma, urinary bladder cancer has become one of the most lethal of the urological neoplasms. In 2018, about 81,190 new cancer cases and 17,240 deaths related to bladder tumor are estimated to be found in the United States 1. Muscle-invasive urinary bladder cancer (MIBC) makes up for about 25% of initially diagnosed bladder carcinoma cases. However, up to 10% to 15% of patients with non-muscle-invasive urinary bladder cancer (NMIBC) will progress to MIBC 2, 3, leading to an increase in the mortality of bladder cancer.

Most of the bladder cancer patients receive diagnostic procedures after certain symptoms, including hematuria, have already appeared. It is estimated that approximately 3% to 15% of the patients with hematuria were finally diagnosed with urinary tract cancer 4-6. As a typical diagnostic analysis of hematuria, cystoscopy has been recommended by the current guidelines, which has a sensitivity of 87% to detect bladder malignant tumor in patients with gross hematuria 7. However, cystoscopy is invasive, which causes pain and discomfort to patients 8.

Fortunately, urinary epigenetic biomarkers, including DNA methylation, have been developed to provide effectual method for detecting bladder cancer 9, 10, based on the theory that epigenetic alterations precede the initial mutations in cancer 11-14. The alterations in the state of DNA methylation, which can be detected prior to oncogenesis, contribute to the development and progress of various cancers. Cancer-associated methylation may act as a proposal of candidate markers 15-18. However, few studies have reported the cancer-specific urinary DNA methylation for bladder in Chinese population.

In this present study, we carried out an evidence-based analysis based on the candidate methylation makers which have been shown to be closely related to bladder cancer in previous studies. Our aim is to evaluate the ability of optimized combination of methylation genes to detect bladder carcinoma in Chinese patients with hematuria.

## Materials and methods

### Patients and samples

A number of 99 Chinese patients with hematuria in Huashan Hospital, Shanghai, China were recruited in our study from 2015 to 2016. None of these patients had any history of urologic neoplasms before. The protocols of our research had been authorized by Institutional Review Board at Huashan Hospital and informed written consent was required from all the participants.

The Cancer Genome Atlas (TCGA) cohort was retrieved from online data repository. A total of 412 bladder cancer patients and 21 matching normal tissue were included in the TCGA cohort with methylation (HM450) beta-values and clinical data.

Urine samples were obtained from these recruited 99 patients before they underwent cystoscopy for diagnostic assessment or treatment, pelleted by centrifugation at 3,000 rpm. The supernatants of the centrifuged samples were discarded, leaving the cell pellets to be washed by 10 ml phosphate buffered saline and then be centrifuged at 3,000 rpm for 10 minutes (min). Supernatant was removed again and the sediments were frozen at -80 °C.

### Identification of candidate methylation markers

Literature search was performed by using PubMed to identify significant methylation genes proved to be closely related to bladder cancer as urine biomarker candidates in previous studies. The search strategy, including “methylation”, “bladder” and “urine”, was applied to PubMed between 2000 and 2016 and found out 135 articles related. To identify strong and solid evidences of candidate methylation markers, only choreographed cohort study or case-control study, including NMIBC (Ta-T1) as a phenotype, with a urinary DNA sample size over 100 was selected in our study. Thirty-eight candidate genes were mentioned in 14 studies, of which 7 genes (*HOXA9*, *ONECUT2*, *PCDH17*, *PENK*,* TWIST1*,* VIM* and *ZNF154*) reported over twice in different studies were finally selected and used for further study. The process of identification of candidate methylation markers was shown in Figure 1.

### DNA isolation and bisulfite conversion

DNA of the urine sediments was isolated by using the QIAamp DNA Micro Kit (Qiagen) according to the manufacturer's recommendations. The Fluorometer (ThermoFisher Scientific) and NanoDrop Microvolume Spectrophotometers were employed to quantify the concentration of DNA. After bisulfite conversion by EZ DNA Methylation-Gold™ Kit (Zymo Research), the DNA was then purified using 30 μl of M-Elution Buffer (Zymo Research) and was frozen at -80 °C.

### Methylation analysis

We performed high resolution melting-curve assays to analyze the methylation level of exon regions or the promoter CpG islands of the selected genes (*HOXA9*, *ONECUT2*, *PCDH17*, *PENK*,* TWIST1*,* VIM* and *ZNF154*) by making the samples situated at 72.0 - 95.0 °C for 15 seconds (sec) and then cooling them to 60.0 °C at the rate of 0.025 °C/sec. They were further melted from 60.0 °C to 95.0 °C by 0.025 °C/sec, sustaining for 15 sec, and cooled to 60.0 °C again at the rate of 1.6 °C/sec. HRM-PCR for cloning was carried out with QuantStudio 7 Flex (Life Technologies of Thermo Fisher Scientific) after a pre-incubation of 10 min at 95 °C. The reactions were then executed for 50 cycles of denaturation at 95.0 °C for 15 sec, annealing at 60.0 °C for 30 sec and extension at 72.0 °C for 15 sec.

Each reaction mixture was designed to be composed of 5 μl of 2×ZymoTaq™ qPCR Premix (Zymo Research), 0.5 μl of LC Green^Plus^ (BioFire Diagnostics), 1 μl of 3μM mixed primers (reverse and forward primer), 1 μl of DNA template and 2.5 μl of nuclease-free water.

The aligned high resolution melting data were exported and processed using a binary system to qualitatively analyze the methylation of the selected genes. Samples with significantly higher value than controls' mean value in the measured methylation were regarded as methylation positive.

### Statistical analysis

Categorical variables were shown as percentage and compared using a Pearson's Chi-square test or a two-tailed Fisher's exact test, as appropriate. Univariate and multivariate binary logistic regression analyses were done to evaluate the association between bladder cancer and each predictor variable. A risk score formula was then developed and calculated by the targeted genes, weighted by their estimated regression coefficients from the multivariable binary logistic regression analyses. Receiver operating characteristic (ROC) curves was used to assess the specificity and sensitivity of bladder cancer prediction on the base of methylation risk score, and area under the curve (AUC) was calculated from the ROC curve. All statistical analyses were performed using SPSS 13.0 (SPSS Inc., Chicago, IL, USA). A *p* value of less than 0.05 (two-sided) was considered to indicate statistical significance.

## Results

Of the 99 participants selected for our research, 18 urine samples were discarded because the DNA yield was too low for accurate methylation analysis. The 81 attainable urine samples from 44 bladder cancer patients and 37 control patients were applied to perform methylation specific high resolution melting-curve (MS-HRM) PCR assay for the detection of bladder cancer. The demographic characteristics of included patients were summarized in Table 1. All bladder cancer cases were diagnosed according to 2004 WHO grading. Among 44 bladder cancer patients in Huashan cohort, 17 (38.6%) patients were diagnosed with high grade disease. While in the TCGA cohort, 388 (94.2%) of the bladder cancer patients were diagnosed with high grade disease. Control patients in the Huashan cohort were diagnosed of benign prostatic hyperplasia, urinary calculi or urinary tract infection.

To explore the association between DNA methylation and bladder cancer, an analysis was further set up to compare the probability of DNA methylation in both bladder cancer and control groups (Fig 2a). We found increased probability of DNA methylation of all the selected 7 genes in bladder cancer group than the control group in Huashan cohort. To verify our results, we further assessed the relationship between DNA methylation beta-values and bladder cancer in TCGA cohort (Fig 2b). Strikingly, remarkable higher DNA methylation beta-values of all the selected 7 genes were displayed in bladder cancer tissues compared with normal bladder tissues, which was consistent with observations in Huashan cohort, which revealed the potential predictive values of the selected 7 genes on bladder cancer.

Logistic regression analyses of 7 targeted genes in Huashan cohort were shown in table 2. In univariate logistic regression analysis, all of the 7 targeted genes were signally connected with bladder cancer. Multivariate logistic regression analysis was then performed to calculate estimated regression coefficients of the 7 selected genes. A risk score formula was then created on the base of the combined methylation expression for bladder cancer prediction, as follows: risk score = (8.919*expression level of *HOXA9*) + (13.513*expression level of *ONECUT2*) + (13.119*expression level of *PCDH17*) + (2.534* expression level of *PENK*) + (1.151*expression level of *TWIST1*) + (0.405*expression level of *VIM*) + (0.306* expression level of *ZNF154*). The methylation expression of methylated genes were defined as “1”, while the methylation expression of non-methylated genes were defined as “-1”.

ROC analysis was carried out to evaluate the specificity and sensitivity of bladder cancer prediction by our risk score in Huashan cohort and TCGA cohort. As shown in Fig. 3a and Fig. 3b, our risk score model could reach notable AUC of 0.894 and 0.851 in respective cohort. Overall multivariate logistic regression analysis also resulted in consistent predictive value of risk score in the two cohorts (Table 3), revealing that our risk score model had highlighted predictive value for bladder cancer diagnosis.

## Discussion

Currently, cystoscopy has been recommended as the standard treatment for diagnosis of bladder cancer. However, not only it is limited to the tumors that can be identified visually, and cystoscopy is also invasive and costly, which can cause discomfort for the patient 7, 8, 19. Considering such high diagnostic costs and high patient burden caused by cystoscopy, some noninvasive molecular tests, including BTA test, NMP22, and cytology, have been developed to try to replace the use of cystoscopy for patients with hematuria. Nevertheless, because of their low diagnostic accuracy, these noninvasive exams fail to be conventionally used in diagnosis and monitoring of bladder cancer 20, 21.

Here, we established a combination methylation assay of *HOXA9*, *ONECUT2*, *PCDH17*, *PENK*,* TWIST1*,* VIM* and *ZNF154*, which had displayed great prediction accuracy of bladder cancer in patients with hematuria by using urine samples. Using our risk score model, the combination of methylation markers performed stably and the bladder cancer could be accurately predicted with a notable AUC of 0.851-0.894. Our result was of great significance since it contributed important approach to develop noninvasive examination thereby reducing the frequency of cystoscopy for patients with hematuria.

Our study had several additional advantages compared to previous studies on urine DNA methylation, where the results were either unverified or had a lower diagnostic power. Firstly, a strict and scientific criterion was conducted to identify the candidate epigenetic markers, so that the strong and solid evidences of candidate markers were guaranteed. Secondly, the result of our study was validated in 412 bladder cancer patients and 21 matching normal tissue from the TCGA cohort with methylation (HM450). This was in line with current research ideas in translational medicine. Besides, the method of methylation, HRM-PCR, was cost-effective and high sensitive compared with other methods in previous studies.

However, there were also several limitations in the current study. Firstly, our research had not reported a certain new gene methylations since the candidate methylation genes were recruited from previous studies. Secondly, the small size in our test series was also a limitation, although the validation series from large sample maybe made up the defection to some extent. A prospective study based on a hematuria cohort with a large sample size should be conducted to validate these findings in the future.

## Conclusion

An assorted methylation detection of *HOXA9*, *ONECUT2*, *PCDH17*, *PENK*,* TWIST1*,* VIM* and *ZNF154* from urinary sample displayed great prediction accuracy of bladder cancer from clinical hematuria patients, which means unnecessary invasive test could be avoided for cancer patients at early stage and during the follow-up after operation. A prospective study in the base of a hematuria cohort with a large sample size is still needed to validate this urinary biomarker combination.

## Figures and Tables

**Figure 1:** Process to identify candidate methylation markers.

**Figure 2:** (**a**) Comparation of the probability of DNA methylation in bladder cancer and non-bladder cancer patients in Huashan cohort. (**b**) Comparation of DNA methylation beta-values of bladder cancer tissues and normal bladder tissues in TCGA cohort. Bca, bladder cancer; non-BCa, non-bladder cancer; ***, P < 0.001; **, P < 0.01; *, P < 0.05.

**Figure 3:** (**a**) Receiver operating characteristic (ROC) analysis of the sensitivity and specificity of bladder cancer prediction by the risk score in Huashan cohort. (**b**) ROC analysis of the sensitivity and specificity of bladder cancer prediction by the risk score in the TCGA cohort. AUC, area under the curve; *CI*, confidence interval.

**Table 1:** Demographic characteristics of including patients

	Huashan cohort				TCGA cohort	
	Bca	non-BCa	*P* value		Bca	Normal tissue
**No. of patients**	44	37			412	21
**Age(yr)**			0.078			
**Mean**	66.0	61.0			75.0	77.4
**Range**	57.3-75.0	51.0-68.3			40.0-98.0	54.0-94.0
**Gender**			1.00			
**Male**	38(86.4%)	32(86.5%)			301(73.0%)	11(52.4%)
**Female**	6(13.6%)	5(13.5%)			107(26.0%)	10(47.6%)
**Unknown**	0	0			4(1.0%)	0
**Tumor Grade**						
**High Grade**	17(38.6%)	**/**			388(94.2%)	**/**
**Low Grade**	21(47.7%)	**/**			21(5.1%)	**/**
**Others**	6(13.6%)	**/**			3(0.7%)	**/**

yr, year; Bca, bladder cancer; non-BCa, non-bladder cancer.

**Table 2:** Univariate and Multivariate logistic regression analysis of 7 methylation assays

	Univariate analysis		Multivariate analysis	
	OR (95% *CI*)	*P* value	OR (95% *CI*)	*P* value
***HOXA9***	8.644 (3.13∼23.874)	0.000032*	8.919(1.99∼39.964)	0.004*
***ONECUT2***	33.833 (7.143∼160.256)	0.000009*	13.513(1.128∼161.832)	0.04*
***PCDH17***	30.625 (6.489∼144.534)	0.000015*	13.119(1.51∼114)	0.02*
***PENK***	36 (4.529∼286.155)	0.001*	2.534(0.146∼43.883)	0.523
***TWIST1***	4.288 (1.665∼11.042)	0.003*	1.151(0.246∼5.374)	0.858
***VIM***	11.071 (3.759∼32.605)	0.000013*	0.405(0.042∼3.929)	0.435
***ZNF154***	4.941 (1.881∼12.977)	0.001*	0.306(0.033∼2.862)	0.299

* indicated significant difference; OR, odds ratio; *CI*, *confidence interval*.

**Table 3:** Multivariate logistic regression analysis of risk score

	Huashan cohort		TCGA cohort	
	OR (95% CI)	P value	OR (95% CI)	P value
Age	0.982(0.932∼1.035)	0.501	0.995(0.951∼1.042)	0.838
Gender	5.328(0.544∼52.227)	0.151	2.135(0.819∼5.57)	0.121
Risk score	1.091(1.048∼1.135)	0.00002*	1.405(1.203∼1.64)	0.000017*

* indicated significant difference; OR, odds ratio; *CI*, *confidence interval*.

## Abbreviations

TURBT: transurethral resection of bladder tumor
TCGA: The Cancer Genome Atlas
ROC: receiver operating characteristic
AUC: area under the curve
MS-HRM: high resolution melting-curve
